The article "Pediatric Residency Training amid the COVID-19 Pandemic: Exploring the Impact of Supervision and Clinical Practice Guidelines on Clinical and Financial Outcomes" was published in 2022. Journal: Comput Math Methods Med.

# Pediatric Residency Training amid the COVID-19 Pandemic: Exploring the Impact of Supervision and Clinical Practice Guidelines on Clinical and Financial Outcomes

**DOI:** 10.1155/2022/2495064

**Published:** 2022-09-13

**Authors:** Anang Endaryanto, Arlina Dewi, Kusbaryanto, Ricardo Adrian Nugraha

**Affiliations:** ^1^Master of Hospital Administration, Universitas Muhammadiyah Yogyakarta, Yogyakarta 55183, Indonesia; ^2^Department of Child Health, Faculty of Medicine Universitas Airlangga, Dr. Soetomo General Academic Hospital, Surabaya 60285, Indonesia; ^3^Department of Cardiology and Vascular Medicine, Faculty of Medicine Universitas Airlangga, Dr. Soetomo General Hospital, Surabaya 60285, Indonesia

## Abstract

**Objective:**

This study is aimed at calculating the magnitude of the effect of clinical practice guidelines (CPG) and supervision in inhibiting the negative impact of the COVID-19 pandemic on clinical and financial outcomes of non-COVID-19 inpatient care by pediatric residents in academic medical center (AMC) hospitals during the COVID-19 pandemic.

**Methods:**

The cohort retrospective study was conducted. This study collected patient data from pediatric residency programs. A research cohort consisted of non-COVID-19 pediatric patients at Dr. Soetomo General Academic Hospital. This study compared the subgroup of patients treated during the pandemic with those treated before the pandemic. The results were analyzed using SPSS 26.0 and Smart-PLS.

**Results:**

There was a 41.4% decrease in pediatric inpatients during the pandemic with an increased severity level and complexity level, a reduction of 7.46% availability of supervisors, an increase of 0.4% in readmission < 30 days, an increase of 0.31% in-hospital mortality, an increase the total costs of care, and a decrease of insurance claim profit. CPG did not moderate the effect of the COVID-19 pandemic on the clinical outcomes (*β* = −0.006, *P* = 0.083) but moderated the financial outcomes (*β* = −0.022, *P* = 0.000), by reducing the total cost of care and increasing insurance claim profit. Supervision moderated the effect of the COVID-19 pandemic on the clinical outcomes (*β* = 0.040, *P* = 0.000) by increasing aLOS and on the financial outcomes (*β* = −0.031, *P* = 0.000) by reducing the total cost of care and increasing insurance claim profit. This study model had a 24.0% variance of explanatory power for clinical outcomes and 49.0% for financial outcomes. This study's structural model effectively predicted clinical outcomes (*Q*^2^ = 0.238) and financial outcomes (*Q*^2^ = 0.413).

**Conclusion:**

Direct supervision inhibited the negative impact of the COVID-19 pandemic on both clinical and financial outcomes of non-COVID-19 inpatient care by pediatric residents, while CPG only inhibited the negative impact on financial outcomes. *Implication of This Study*. In a disaster, the availability of CPG and direct supervision makes AMC hospitals able to inhibit the negative impact of disasters on clinical and financial outcomes.

## 1. Introduction

The COVID-19 crisis has seriously impacted the academic medical center (AMC) hospital in the clinical, financial, and health education aspects [1]. Dr. Soetomo General Academic Hospital is an AMC hospital and a national referral tertiary referral hospital with the largest number of beds (1670 beds) and the largest number of residents (1890 medical doctors) in Indonesia. In including residents to manage patients, hospitals must apply high-value, cost-consciousness care so that specialists or senior medical doctors must supervise there. High-value cost-consciousness care is easier to implement in AMC hospitals if they implement clinical practice guidelines (CPG), especially for diseases categorized as “high volume,” “high risk,” “high cost,” and “high variability” [2, 3], have an active supervisor medical doctor, and supported by other health professionals in sufficient numbers [4, 5]. The unavailability of CPG and the lack of support from other health workers, especially nurses, will threaten the high-value, cost-conscious care [6–8]. CPG availability is also highly dependent on the speed of adjustment to changes in the profile of patient visits to the hospital [4, 5] because the need for types of CPG can change in a disaster or pandemic condition [3, 9]. Changes in the profile of hospital visits are due to restrictions on admitting patients for nonemergency cases, fear of patients being infected in hospitals, and restrictions on social interaction by the government [10–18].

The quality of patient care is influenced by the presence and compliance of CPG [8, 19, 20]. The complexity of the diagnosis influences CPG availability for each diagnosis. Changes in the complexity of patients raise the need to create new CPGs. However, referring to the results of Cabana et al.'s research, it turns out that 15.7% of medical doctors do not realize that CPG is important, and 10.6% of medical doctors do not know that there is CPG for the case they are being treated in AMC hospital, and even 6.3% of medical doctors disagree that patient care is regulated by CPG [6]. CPG increases the speed of decision-making and execution by a resident when the supervisor medical doctor cannot be present in person in the AMC hospital [8, 19, 20]. Inappropriate use and availability of health service resources in hospitals are one of the significant impacts of the pandemic [21–23]. The pandemic has caused most hospitals to experience disruptions in the availability of health care resources. In AMC hospitals, care by residents without supervision can be a cause of inappropriate and inaccurate use of health care resources, such as supporting examinations and administering drugs [24]. The speed of execution of medical doctors' decisions by nurses is influenced by the direct presence of nurses in hospitals [25–27]. During the pandemic, the presence of health workers is reduced due to infection, death, and isolation [28–33].

The impact of disruption of health services on pediatric patients due to the COVID-19 pandemic in the future must be anticipated, mitigated, and minimized based on valid evidence. In addition, health care methods for pediatric patients that have been proven effective in dealing with pandemics/disasters must be applied so that we are better prepared to face another pandemic or when we face certain circumstances with insufficient resources as happened during a pandemic.

The main contribution of this research is to provide answers based on scientific evidence on whether increased supervision of residents and the existence of CPG can be a solution to disrupted play in AMC hospitals due to the scarcity of resources for specialist doctors and nurses during a disaster.

We are interested in exploring pediatric inpatient services during the COVID-19 pandemic because of the many challenging aspects of the COVID-19 pandemic in pediatric care, including reducing the number of patients with increased complexity, burden, and pressure on pediatric residents in implementing “high value and cost consciousness care” [34]. Hypothesis development: from the many references and evidence above, we propose 20 hypotheses as follows (Figure 1): Hypothesis 1 (H1): COVID-19 pandemic has a significant influence on clinical outcome; Hypothesis 2 (H2): COVID-19 pandemic has a significant impact on the financial outcome; Hypothesis 3 (H3): COVID-19 pandemic has a significantly positive impact on patient condition; Hypothesis 4 (H4): COVID-19 pandemic has a significantly negative impact on nurse adequacy; Hypothesis 5 (H5): COVID-19 pandemic has a significantly negative impact on supervision; Hypothesis 6 (H6): COVID-19 pandemic has a significantly negative impact on CPG; Hypothesis 7 (H7): the patient's condition has a significantly positive influence on supervision; Hypothesis 8 (H8): supervision has a significant effect on clinical outcome; Hypothesis 9 (H9): supervision has a significant impact on the financial outcome; Hypothesis 10 (H10): CPG has a significant impact on clinical outcome; Hypothesis 11 (H11): CPG has a significant impact on the financial outcome; Hypothesis 12(H12): the patient's condition has a significant impact on the clinical outcome; Hypothesis 13 (H13): the patient's condition has a significant impact on the financial outcome; Hypothesis 14 (H14): nurse adequacy has a significant impact on clinical outcome; Hypothesis 15 (H15): nurse adequacy has a significant impact on the financial outcome; Hypothesis 16 (H16): clinical development has a significant impact on the monetary outcome; Hypothesis 17 (H17): CPG moderated the effect of the COVID-19 pandemic on the clinical outcomes; Hypothesis 18 (H18): supervision moderated the impact of the COVID-19 pandemic on the clinical outcomes; Hypothesis 19 (H19): CPG moderated the impact of the COVID-19 pandemic on the financial outcomes; Hypothesis 20 (H20): supervision moderated the impact of the COVID-19 pandemic on the financial outcomes.

This study is aimed at calculating the magnitude of the effect of supervision and CPG in inhibiting the negative impact of the COVID-19 pandemic on clinical and financial outcomes of pediatric inpatient care by pediatric residents in academic medical center (AMC) hospitals during the COVID-19 pandemic.

In this paper, we will inform the method we used to calculate the magnitude of the effect of supervision and CPG in preventing the negative impact of the COVID-19 pandemic on pediatric residents' clinical and financial outcomes of pediatric hospitalization. In the chapter on research results and discussion, we report the impact of the COVID-19 pandemic on AMC hospital on patient care resources and outcomes in clinical and financial aspects, measurement model assessment, results of structural modeling of COVID-19 pandemic in AMC hospital, the role of CPG and supervision, implementation of CPG with supervision, the main finding, limitations, and strengths of the study.

## 2. Materials and Methods

### 2.1. Study Design, Sample Size, Data Collection, and Data Source

The cohort retrospective study was conducted. This study collected patient data from pediatric residency programs of the Faculty of Medicine Universitas Airlangga. A research cohort consisted of non-COVID-19 pediatric patients at Dr. Soetomo General Academic Hospital who were paid using National Health Insurance. This study compared the subgroup of patients treated during the pandemic with those treated before the pandemic. Data were collected retrospectively for 24 months before the pandemic (1 March 2018 to 29 February 2020) with 24 months during the pandemic (March 1, 2020, to February 29, 2022). The study was conducted according to the guidelines of the Declaration of Helsinki and approved for exempt review by the Research Ethics Committee of Dr. Soetomo General Academic Hospital, Surabaya, Indonesia (2022), with reference number 0383/KEPK/III/2022. The sample of this research is the total sample. The entire selection of non-COVID-19 hospitalized pediatric patients 24 months before and 24 months during the pandemic were 35,256 cases. When calculated statistically, which provides sufficient power (*β* = 90%), with a Minimum Detectable Effect (MDE) of 5%, with a level of significance (*α*) 5%, the minimum sample size has been reached.

### 2.2. Variables

The independent variable was the COVID-19 pandemic. The dependent variable was the clinical outcome of care (readmission < 30 days, average length of stay, and in-hospital mortality) and financial outcome of care (total costs of care, hospital revenue, and insurance claim profit). The intervening variables were nurse adequacy, disease severity and complexity, CPG (CPG availability, CPG compliance, and CPG coverage), and supervision (supervisor availability, supervision method, and consultant supervision). This study explored the supervision and CPG moderating variable to calculate the role of supervision and CPG in inhibiting the negative impact of the COVID-19 pandemic on clinical and financial outcomes of pediatric inpatient care by pediatric residents in academic medical center (AMC) hospitals during the COVID-19 pandemic. In this study, all items of variables were in the reflective measurement [35].

Nurse adequacy was the suitability of the number of nurses in percent compared to the number of nurses who should be in the treatment room according to the number of patients and the level of emergency (low care, high care, and intensive care). Disease severity was classified into mild, moderate, and severe disease severity based on INA-CBGs (Indonesia Case-Based Groups) version 4.0 [36]. The complexity of the disease was reflected by the number of diagnoses (comorbidities) in the patient. CPG includes aspects of CPG availability which measures the percentage of CPD availability based on the patient's diagnosis (ICD X), CPG compliance which measures the percentage of resident or supervisor compliance with CPG, and CPG coverage which measures the rate of the presence of CPG for all established diagnoses. Meanwhile, the supervision assessed includes supervisor availability which measures the percentage of supervisor's presence at the hospital, supervision method, which measures the rate of direct supervisor's presence in front of the patient's bed, and the percentage of consultant supervisor's attendance which measures the attendance level of consultant medical doctors across subspecialists.

Readmission less than 30 days was the percentage of patients readmitted less than 30 days from discharge from the hospital. Length of stay (LOS) is the duration (in days) of care of the patient treated for 1 episode of treatment. In-hospital mortality is the incidence of death in hospitalization. Total costs of care based on hospital rates were the full-service costs, including nonsurgical and surgical procedures, consultations, experts, nursing services, radiological examinations, laboratory examinations, blood services, medical rehabilitation, accommodation and rooms, use of drugs (symptomatic, antibiotics, drugs, chronic disease, and chemotherapy), medical devices, consumables, and equipment rental. Hospital revenue was the hospital's total income from claim fees paid to hospitals by National Health Insurance. Insurance claim profit was a profit from insurance claims after deducting care costs.

### 2.3. Statistical Analysis

We used SPSS version 26 to test the normality distribution of all variables and compare values for all variables during the pandemic to before. The comparison test uses an independent *T*-test if the data were normally distributed and uses the Mann–Whitney test or the Kruskal-Walis test (depending on the data being numerical or categorical) if the data is not normally distributed.

Furthermore, to prove the hypotheses in our structural model (Figure 1), we use Structural Equation Modeling (SEM). If the data were normally distributed, we used Covarian Based SEM (CB-SEM) with AMOS software, and if the data was not normally distributed, we used Partial Least Squares SEM (PLS-SEM) with Smart-PLS software. We used AMOS or Smart-PLS software (the choice depends on the distribution of our research data) to test all the hypotheses in Figure 1.

Firstly, we measured Confirmatory Factor Analysis (CFA) with unidimensionality for each scale and reliability-validity of each construct. We look at the unidimensionality for each scale with factor loading, and if it shows a value less than 0.500 [37], we will remove it. Because the items from our variable (construct) were reflective, the reliability indicators were loading factors, Cronbach's alpha, composite reliability, and average extracted variance (AVE). Construct reliability was achieved when the factor loading value was greater than 0.700 [38], Cronbach's alpha, and composite reliability were equal to or greater than 0.600. The validity indicators were average extracted variance (AVE), Fornell–Larcker criteria (square root of the AVE for each variable was higher than the variance of the variable divided by other variables) [38], Heterotrait–Monotrait Ratio of Correlations by Henseler [39] for discriminant validity, and cross loading factors. Validity was achieved when the mean of extracted variance (AVE) for convergent validity was higher than 0.500 [38], Heterotrait–Monotrait Ratio of Correlations (HTMT) value was less than 0.900 [40]. Cross factor loading of items must be higher with each variable than with other variables. After that, we also had to assess whether there was a collinearity problem in the model by looking at the correlation matrix and variance inflation factor (VIF). If the value of VIF was less than 3.30 [37], there was not a collinearity problem in the model. The general threshold of VIF was 5 [38]. If there were no problems with multicollinearity, PLS-SEM was better for estimating the path coefficients among the latent variables of the structural model [41]. To assess the explanatory power of the structural model, we measured *R*^2^ values. *R*^2^ values 0.75, 0.50, and 0.25 were considered substantial, moderate, and mild, respectively [42]. To assess individual predictors and their role in the model, we measure effect size (*f*^2^). The *f*^2^ values of 0.35, 0.15, and 0.02 refer to the large, medium, and small effect of an independent variable [43]. To assess and predict relevancy and accuracy in the model, we measure *Q*^2^. *Q*^2^ value was greater than zero indicating a model relevant and accurate [42].

## 3. Results and Discussion

### 3.1. Impact of COVID-19 Pandemic on AMC Hospital

Table 1 shows that during COVID-19 pandemic (from March 1, 2020, to February 29, 2022) compared to before (from 1 March 2018 to 29 February 2020), there were 41.4% decreasing in pediatric inpatient, increase 0.44 years in the average inpatient age (*P* = 0.000), increase 0.08 of severity level and 0.31 of complexity level of the disease (*P* = 0.000), increase of medical cases by proportion (0.9%) and decrease by number (7005 cases) (*P* = 0.045), decrease of surgical cases both proportion (by 0.9%) and number (1730 cases) (*P* = 0.042), increase 2.62% of CPG availability (*P* = 0.000), decrease 3.99% direct supervision and decrease 7.46% availability of supervisors (*P* = 0.000), increase supervision by consultant (1.34%) (*P* = 0.000), decrease 21.9% adequacy of nurses (*P* = 0.000), increase 0.4% readmission < 30 days (*P* = 0.000), increase 0.31% in-hospital mortality (*P* = 0.000), increase (IDR × 1,000) 3,937.4 of the total costs of care/patient (*P* = 0.000), slight increase (IDR × 1,000) 524.8 of hospital revenue/patient (*P* = 0.000), and significant decrease (IDR × 1,000) 3,412.6 of insurance claim profit/patient (*P* = 0.000).

A decrease in inpatient visits for pediatric patients (Table 1) can be caused by a reduction in the provision of health services, insecurity, restrictions on public activities, high-risk communication, and the fear of being exposed to COVID-19 infection through interactions with each other, which also makes people reluctant to leave their homes and seek routine health care [44–46]. The results of the ECIEN-2020 study also showed that the COVID-19 pandemic, especially during the lockdown, led to a decrease in the number of visits to the pediatric ER and admissions of pediatric patients to hospital inpatients an increase in the severity and complexity of respiratory illnesses [47]. The high complexity of inpatient and urgent/emergency care for non-COVID-19 patients has also been reported in many previous studies [47–51]. Several previous studies also showed that the COVID-19 pandemic affected pediatric surgery services [52–55].

The decrease in the number of direct supervision and the adequacy of nurses (Table 1) due to COVID-19 infection is a very detrimental impact of the pandemic. This condition can be influenced by the home or hospital environment that does not create social distance and pays less attention to fundamental health problems. The results of numerical simulation research for optimal control strategies in Iran and Japan show that by creating social distance and paying attention to basic health problems, disease prevalence is controlled [56]. In a hospital setting, asymptomatic infections play an important role in developing infections, so educating all health workers on avoiding contact with these individuals [57] is necessary.

The decrease in nurse adequacy (Table 1) occurred not only during a pandemic but also in other conditions. A study informs that a reduction of the adequacy of nurses can occur outside of working hours. Of patients, more than a third was treated outside of working hours. Out-of-work care—evenings, weekends, and holidays—is characterized by a decrease in the adequacy of nurses and other staff and a reduction in the availability of certain diagnostic and support services [58]. In addition, the availability of nurses with appropriate expertise also determines the outcome of medical services in hospitals [59].

Decreasing LOS involves controlling for many factors. To reduce their caseload, residents tend to lower their LOS, with the negative impact of increasing less than 30 days of readmission. However, the facts show that patients admitted to AMC hospitals have a much shorter LOS, fewer consultants, and lower direct care costs than non-AMC hospitals. It is recognized that hospital workloads may have a negative impact on clinical and financial outcomes. However, the study at AMC hospital showed that outcomes for in-hospital mortality and less than 30 days readmission did not appear to be affected by workload [1]. There is a relationship between patient mortality at AMC hospital and the involvement of hospital leaders, including clinical department heads. In the AMC hospital, without the participation of the clinical department chair, the mortality reduction performance did not improve [58]. One of the possible reasons was the resident's natural desire to reduce their caseload. Besides, the pandemic period has made parents want their children to get out of the hospital faster [1].

### 3.2. Measurement Model Assessment

Because the data distribution of the dependent variable was not normally distributed, we used Partial Least Squares (PLS-SEM) with Smart-PLS software to assess the measurement model and the structural model of the conceptual framework. Items of supervisor consultant, CPG availability, readmission less than 30 days, in-hospital mortality, and hospital revenue were removed from the model (Table 2) due to the factor loading value being less than 0.700. Construct reliability was achieved because the factor loading value was more significant than 0.700 [38], and Cronbach's alpha and composite reliability were equal to or greater than 0.600 (Table 3). Validity was achieved due to the mean of extracted variance (AVE) for convergent validity was higher than 0.500, Heterotrait–Monotrait Ratio of Correlations (HTMT) value was less than 0.900 (Table 4), cross factor loading of items was higher with each variable than with other variables (Table 5), and the correlation matrix and variance inflation factor (VIF) was less than the general threshold of VIF (Table 6). Because there were no problems with multicollinearity, the structural model was better for estimating the path coefficients (Table 7). The measurement of our model meets all the criteria for a good fit and is suitable for Hypotheses testing (Table 7). As shown in Table 8, this study model had a 24.0% (*R*^2^ = 0.240) or mild variance of explanatory power for clinical outcomes and 49.0% (*R*^2^ = 0.490) or moderate variance for financial outcomes. This study's structural model effectively predicted clinical outcomes (*Q*^2^ = 0.238) and financial outcomes (*Q*^2^ = 0.413).

### 3.3. Results of Structural Modeling of COVID-19 Pandemic in AMC Hospital

About the COVID-19 pandemic, from the structural model (Figure 2 and Table 7), our study showed that COVID-19 pandemic had the following: (1) direct effect on a pediatric patient's condition (*β* = 0.069, *P* = 0.000) increases severity and complexity; (2) direct effect on decreasing nurse adequacy (*β* = −0.621, *P* = 0.000); (3) no direct effect on CPG (*β* = −0.006, P = 0.262); (4) direct effect on supervision (*β* = −0.103, *P* = 0.000), by decreasing direct supervision and supervisor availability; (5) indirect effects on clinical outcome (*β* = −0,041, *T* = 8.825, *P* = 0.000) by decreasing aLOS; and (6) the indirect effect on financial outcomes (*β* = 0.069, *P* = 0.000) by increasing the total cost of care and decreasing the insurance claim profit.

This finding (Figure 2 and Table 7) implies that residents need to be made aware that runaway medical costs will threaten the accessibility and affordability of the health care system. Thus, insight into high-value, cost-conscious care should also be emphasized in residents who, in the past, focused solely on clinical outcomes [59]. There has been little emphasis on high-value, cost-consciousness care in the resident education process in the past. To enhance learning, residents should feel free to ask their supervisors critical questions and discuss dilemmas and differing beliefs regarding high-value, cost consciousness care. For this reason, both the resident education program and current departmental policies must contribute to the high-value, cost consciousness care learning [59].

The supervisor is responsible for controlling 80% of health expenditures. Our study showed that supervision had a significant impact on the financial outcome (*β* = −0.150, *P* = 0.000) by reducing the total cost of care and increasing insurance claim profit; therefore, the supervision of residents plays a significant role in achieving a waste reduction in hospitals. Residents should be trained in high-value, cost-conscious care earlier to reduce waste in the future. Waste in health services reaches 20%. Reducing waste will increase profits [59]. It is known that residents are often unaware of the actual costs of care, and few residency programs have a formal curriculum in high-value, cost-conscious care. The data show that the extravagant behavior of the residents persists, and it results from the practice environment in the hospital.

### 3.4. The Role of Clinical Practice Guidelines (CPG)

About CPG, from the structural model (Figure 2 and Table 7), our study showed that (1) COVID-19 pandemic had no direct effect on CPG (*β* = −0.006, *P* = 0.262); (2) CPG significantly impacted clinical outcomes (*β* = −0.078, *P* = 0.000) by decreasing aLOS; (3) CPG significantly impacted the financial outcome (*β* = −0.069, *P* = 0.000) by reducing the total cost of care and increasing insurance claim profit; (4) CPG did not moderate the effect of the COVID-19 pandemic on the clinical outcomes (*β* = −0.006, *T* = 1.735, *P* = 0.083); (5) CPG moderated the impact of the COVID-19 pandemic on the financial outcomes (*β* = −0.022, *T* = 9.376, *P* = 0.000) by reducing the total cost of care and increasing insurance claim profit; and (6) CPG had a significant effect only on financial outcomes (*f*^2^ = 0.009). Preparation of CPG is also associated with improved patient satisfaction and increased implementation of surgical procedures by residents with low complication rates. CPG implementation includes more about procedural actions, the equipment used, and the cost of care [60]. Feedback on CPG implementation and resident performance will improve CPG compliance. A previous study found that CPGs did not significantly affect clinical outcomes [61]. This finding is similar to our result (Figure 2 and Table 7), showing that CPG did not moderate the effect of the COVID-19 pandemic on the clinical outcomes (*β* = −0.006, *P* = 0.083). However, CPG still governs the best practice safety process measures.

Complications due to medical procedures are the second most common cause of side effects among hospitalized pediatric patients. To increase the safety of the action procedure, CPG is required. However, formal procedural resident supervision by experienced supervisors performing bedside medical procedures is required. The results of previous studies inform the medical education community that the development of the CPG did not ensure that residents' chances of gaining hands-on procedural experience would increase. For this reason, simulation training is to complement (not replace) bedside training with direct supervision so that procedural skills are better and safer [61]. CPGs help medical doctors determine the best a patient treatment for a particular medical condition but are not designed to take each patient's unique needs into account. CPG standardizes medical practice according to scientific principles or the best available evidence of effectiveness. By reducing uncertainty, CPG minimizes variation in medical practice, thereby improving outcomes in patient care. In two systematic reviews of the literature, it was found that lack of knowledge and belief in CPG was a significant cause of nonadherence [62].

Our study found that the effect of the COVID-19 pandemic on increasing total cost of care and decreasing insurance claim profit can be inhibited by CPG (Figure 2 and Table 7, hypothesis 19); once again, residents must be made aware that uncontrolled medical expenses will threaten the health of the pocket home business. Insights into high-value, cost-conscious care should also be emphasized to residents. Education residents today are faced with the difficult task of producing medical doctors who are high-value, cost-conscious care-oriented [59]. Exactly why experts are more likely than beginners to deviate from CPG is unclear. One possibility is that, as medical doctors become more skilled, medical doctors move from an analytical approach to an experience-based process. Educational strategies need to be differentiated for medical doctors who are experts and beginners. For specialists, judicious deviation from CPG concerning individual patient circumstances is not only acceptable but also to be expected. [62].

Although CPG is evidence-based, clinical management decisions by clinicians may be influenced by other contextual factors. A drawback of CPG is that in the patient context, particularly aspects of the context that are personal or “nonmedical” (i.e., social) receive relatively less attention than aspects of scientific evidence. Interventions that integrate patient contextual factors into clinical management decisions in resident education can increase cognitive load and result in less-than-optimal learning. The CPG was developed to assist clinicians in determining the best treatment for a patient. However, it was not designed to consider the individual patient's unique needs. One study showed that clinicians were less likely to follow CPG recommendations in the presence of contextual factors than without contextual factors (56% versus 80%, respectively; odds ratio [OR] = 0.32, 95% [CI] = [0.17 − 0.53], *P* < 0,001). Contextual factors include patient learning activities, proximity to care, treatment expectations, and factors related to home life [62].

Effective collaboration among health care team members was crucial; residents often felt pressured following perceived low-value recommendations from consultants [63]; in the absence of contextual factors, expert physicians and novice physicians were equally likely to adhere to the CPG (80% for expert versus 79% for novice physician, OR = 1.05, 95% CI = [0.59, 1.8], *P* = 0.85). A patient's context influences how physicians manage care, even when CPGs are available and known. The previous study does not support the hypothesis that adherence is related primarily to physicians' knowledge of CPGs. Despite this demonstrated familiarity, management decisions deviated from CPGs more often in the presence of a contextual factor. These observations imply that the “lack of adherence” among physicians may not be a function of their level of CPG knowledge but their sensitivity to each patient's unique needs. While based on the best available evidence, clinical management decisions are tailored according to the physician's perception of potential benefits given the whole experience of the patient [62].

### 3.5. The Role of Supervision

Regarding supervision from the structural model (Figure 2 and Table 7), our study showed the following: (1) COVID-19 pandemic significantly impacts supervision (*β* = −0.103, *P* = 0.000); (2) supervision significantly impacted clinical outcomes (*β* = −0.118, *P* = 0.000) by decreasing the average LOS; (3) supervision significantly impacted the financial outcome (*β* = −0.150, *P* = 0.000) by reducing the total cost of care and increasing insurance claim profit; (4) supervision moderated the effect of the COVID-19 pandemic on the clinical outcomes (*β* = 0.040, *T* = 8.825, *P* = 0.000) by increasing the average LOS; (5) supervision moderated the impact of the COVID-19 pandemic on the financial outcomes (*β* = −0.031, *T* = 6.386, *P* = 0.000) by reducing the total cost of care and increasing insurance claim profit; (6) supervision had a strong effect only on clinical outcomes (*f*^2^ = 0.017); (7) the impact of the COVID-19 pandemic on reducing average LOS was complementary to other variables (patient's condition and supervision); and (8) the severity and complexity of the disease increased direct supervision (*β* = 0.220, *P* = 0.000).

Supervisors must be better prepared to teach and set an example in high-value, cost-conscious care to educate residents better. Unfortunately, the data show that preparation for this is lacking. We must intervene to educate future medical doctors on the cost of care during residency education [1]. Most of the supervision in clinical education is directed at identifying the patient's condition and providing the “best” therapy for the patient's clinical condition. At the same time, CPG tends to strengthen the rationale for choosing a treatment. On the one hand, supervision supports “patient-centered care” and involves the patient in decision-making; on the other hand, optimal treatment is a direct consequence of scientific evidence implemented in the CPG [62].

For over a century, direct supervision (a bedside round process) in which supervisors and residents discuss inpatient conditions and treatment plans in front of patients has been the ideal learning method in hospitals. A 2009 study showed that only 17% of resident supervision occurred in patients' rooms at the bedside. Restrictions on resident working hours, and increasing reliance on technology, have caused medical doctors and senior residents to seek other forms of learning that are considered more efficient, namely in the conference room. Despite the rhetorical and theoretical merits of direct supervision (a bedside round process), recent research has shown that resident supervision occurring at the bedside in patient rooms is decreasing. Yet, since the mid-20th century, the bedside round process was the norm. Today, experts and leaders want clinical learning methods to return to the bedside round process. Direct supervision (bedside round process) allows residents to develop their skills, practice teamwork, and communicate with patients and all hospital staff for patient-centered care [64].

### 3.6. Implementation of CPG with Supervision

Implementation of CPG alone had no impact on clinical outcomes. Still, the implementation of CPG by residents with supervision by senior medical doctors had a much lower procedural failure rate (4.2% vs. 7.2%, *P* = 0.020) [60]. With supervised CPG implementation, appropriate ultrasound guidance was higher (96.8% vs. 90.0%, *P* = 0.004) and lower femoral CVC rates (10.5% vs. 17.3%, *P* = 0.020). The direct supervision performed at AMC hospital on pediatric residents is safer than previously thought. Cost savings occurred with a greater opportunity when performing a medical procedure based on the CPG supervisor was present (26.6% vs. 7.6%, *P* < 0.0001) [61]. Feedback on CPG implementation and residents' performance will increase residents' compliance with CPG [65]. In implementing CPG, performing bedside medical procedures without supervision by a senior medical doctor did not improve clinical outcomes but can still enhance financial outcomes [61]. In other words, as we found from our research (Figure 2 and Table 7), supervision and CPG reduce the total costs of care that increased during the COVID-19 pandemic and increase insurance claim profit that decreased during the COVID-19 pandemic. This study proves that if the supervision of residents occurs at the bedside in the patient's room, high-value cost-consciousness care is easier to achieve (Tables 1 and 7 and Figure 2).

On the other hand, some residents also questioned the benefits of the bedside round learning process and whether bedside rounds could continue to be considered a standard of educational practice. However, almost all residents believe that the learning process at the bedside positively influences resident behavior in providing health care in hospitals [64]. The supervisor was an effective role model for residents in making complex clinical decisions and allowed them to pursue their preferred plans [59]. In several academic hospitals, the implementation of supervision and CPG was developed through a bedside round process to improve patient safety and the quality of resident education [61]. Therefore, the introduction of CPG and supervised bedside rounds should be given up front during resident orientation before working in AMC hospitals, including diagnostic and treatment algorithms [1].

### 3.7. The Main Finding

The most important result of this paper is to find out how big the role of supervision and CPG is when health human resources are scarce, especially doctors and nurses, during a pandemic. The main finding of this study is that direct supervision inhibited the negative impact of the pandemic on both clinical and financial outcomes of non-COVID-19 inpatient care by pediatric residents. In contrast, CPG was only inhibited on financial outcomes. Based on the facts, our research has proven that the COVID-19 crisis has seriously impacted the academic medical center (AMC) hospital in the clinical, financial, and health education aspects (Table 1, Figure 2, and Table 7). This research's novelty is quantifying the effect of CPG and supervision on medical services in AMC hospitals by pediatric residents on clinical outcomes and financial outcomes in times of resource scarcity. Previous literatures, which also discussed Supervision and/or CPG [1, 60–64, 66–72] have not calculated how big the “effect size” of Supervision and CPG is on clinical outcomes and financial outcomes in conditions of resource scarcity.

The COVID-19 pandemic also has triggered significant changes in medical education. Effective learning designs need to be developed and implemented to address COVID-19-related barriers in resident education to help educators turn the COVID-19 crisis into opportunities for positive and sustainable change. Supervision with a practical design enables residents to make complex clinical decisions and develop their competence in the high-value, cost-conscious care [69]. It is not surprising that today's academic lecturers have difficulty teaching high-value, cost consciousness care, as they were previously untrained [59]. The results of this study imply that, in a disaster, the availability of CPG and direct supervision makes AMC hospitals able to inhibit the negative impact of disasters on clinical and financial outcomes.

What is not available in previous papers [1, 60–64, 66–72], is that this paper provides information on the right solution for AMC hospitals forced to experience resource scarcity. The impact of disruption of health services on pediatric patients due to the COVID-19 pandemic in the future must be anticipated, mitigated, and minimized based on valid evidence. In addition, health care methods for pediatric patients that have been proven effective in dealing with pandemics or disasters must be studied and applied so that we are better prepared when facing another pandemic or certain circumstances with insufficient resources similar to the pandemic.

### 3.8. Limitations and Strengths of the Study

The limitations of this research are the following: (1) the design used is retrospective; there are limitations to this retrospective study; (2) the research subjects only came from one hospital (the largest AMC hospital in Indonesia); and (3) data is only taken from pediatric patients financed by national health insurance. To consolidate our findings, further prospective multicenter studies should include more hospitals. The strengths of this research are the following: (1) the number of subjects observed was quite large, comparing the pandemic conditions with the previous one with a long observation period (24 months) before the pandemic and 24 months during the pandemic; (2) use path analysis with a structural equation model (SEM) to explore the relationship between research variables. PLS-SEM is an appropriate, robust, and powerful tool [73, 74]; and (3) our study found that the *Q*^2^ value was more significant than zero (Table 8). Information in Table 8 indicating the relevance and accuracy of path model predictions is acceptable for certain variables. Therefore, this model effectively predicts clinical outcomes (*Q*^2^ = 0.238) and financial outcomes (*Q*^2^ = 0.413).

## 4. Conclusions

This study proves that direct supervision contributes to inhibiting the negative impact of the COVID-19 pandemic on the clinical and financial outcomes of non-COVID-19 inpatient care by pediatric residents. On the other hand, CPG only contributes to financial results.

We recommend a multicenter study on the impact of supervision and clinical practice guidelines on clinical and financial outcomes at AMC hospital to continue this research. In addition, we recommend further research to evaluate the impact of supervision and clinical practice guidelines on conditions where AMC hospital's resources routinely experience a decline in services outside of working days and outside working hours. Information from this research can improve the quality and safety of services under these conditions.

## Figures and Tables

**Figure 1:** Hypothesis development.

**Figure 2:** Result of the structural modeling.

**Table 1:** Characteristics of pediatric patients based on age and sex, case distribution, conditions at admission, adequacy of nurses, CPG, supervision, and outcomes.

Variables	Distribution of pediatric inpatient (*n* = 35,216)					Difference
	Before pandemic (*n* = 22,211)		During pandemic (*n* = 13,005)		*P*	
	*n*	(%)	*n*	(%)		
Sex, male, *n* (%)	9508	(42.8)	5101	(39.2)	0.000	-4407
Case distribution						
Medical, *n* (%)	17,676	(79.6)	10,671	(80.5)	0.045	-7,005
Mix medical-surgical, *n* (%)	1097	(4.9)	626	(4.9)	0.598	-471
Surgical, *n* (%)	3438	(15.5)	1708	(14.6)	0.042	-1730

	Mean	SD	Mean	SD	*P*	Difference
Age (years), mean (SD)	6.3	(5.85)	6.8	(5.92)	0.000	0.44
Patient's condition						
Severity level, mean (SD)	1.8	(0.83)	1.9	(0.83)	0.000	0.08
Complexity level, mean (SD)	2.9	(2.03)	3.2	(2.30)	0.000	0.31
Clinical practice guidelines (CPG)						
% CPG availability, mean (SD)	26.2	(43.95)	28.8	(45.27)	0.000	2.62
% CPG compliance, mean (SD)	19.2	(39.40)	18.4	(38.75)	0.058	-0.82
% CPG coverage, mean (SD)	15.2	(30.74)	15.9	(30.45)	0.060	0.64
Supervision						
% direct supervision method, mean (SD)	75.1	(43.25)	71.1	(45.33)	0.000	-3.99
% supervisor availability, mean (SD)	84.8	(27.61)	77.3	(30.47)	0.000	-7.46
% consultant supervision, mean (SD)	85.7	(35.01)	87.1	(33.57)	0.000	1.34
% nurse adequacy, mean (SD)	83.6	(9.27)	61.7	(18.33)	0.000	-21.93
Clinical outcome						
% readmission < 30 days, mean (SD)	6.3	(5.85)	6.8	(5.92)	0.000	0.44
Average length of stay (days), mean (SD)	9.0	(9.95)	8.9	(10.02)	0.742	-0.1
% in hospital mortality, mean (SD)	2.9	(2.03)	3.2	(2.30)	0.000	0.31
Financial outcome (× 1,000 IDR)						
Total costs of care, mean (SD)	12.021	(21,163.2)	15,59.1	(29,049.6)	0,000	3,937.4
Hospital revenue, mean (SD)	12.186	(16,647.9)	12,711.7	(17,306.9)	0,005	524.8
Insurance claim profit, mean (SD)	165	(15,764.3)	-3,247.4	(22,085.8)	0,000	-3,412.6

**Table 2:** Construct and items construct descriptive statistic.

No.	Constructs	Items of constructs	Mean	SD	1st loading factor	2nd loading factor
1	Pandemic status	Pandemic status	0.37	0.48	1.000	1.000

2	Patient's condition	(1) Severity	1.84	0.83	0.816	0.986
		(2) Complexity	3.03	2.14	0.915	0.989

3	Supervision	(1) Supervision method (%)	73.6	44.07	0.983	0.986
		(2) Supervisor availability (%)	82.0	28.92	0.986	0.989
		(3) Supervision by consultant (%)	86.2	34.48	0.038	Removed

4	CPG	(1) CPG availability (%)	27.1	44.46	0.521	Removed
		(2) CPG compliance (%)	18.9	39.16	0.866	0.988
		(3) CPG coverage (%)	15.5	30.63	0.726	0.827

5	Nurse adequacy	Nurse adequacy (%)	75.5	17.04	1.000	1.000

6	Clinical outcome	(1) Readmission < 30 days (%)	8.5	7.93	0.330	Removed
		(2) aLOS (days)	9.0	9.98	0.875	1.000
		(3) In-hospital mortality (%)	7.5	2.63	0.536	Removed

7	Financial outcome (× IDR 1,000)	(1) Total cost of care	13,475.7	24,447.8	1.000	0.944
		(2) Hospital revenue	12,380.7	16,895.7	0.667	Removed
		(3) Insurance claim profit	-1,095.0	18,427.3	-0.709	-0.911

**Table 3:** Reliability and validity results.

Constructs	Reliability			Convergent validity (AVE) and discriminant validity (square root of AVE)											
	Cronbach's alpha	rho_A	Composite reliability	Average variance extracted (AVE)	Clinical outcome	Clinical practice guidelines (CPG)	Financial outcome	Nurse adequacy	Pandemic status	Pandemic∗CPG (CO)	Pandemic∗CPG (FO)	Pandemic∗ supervision (CO)	Pandemic∗supervision (FO)	Patient's condition	Supervision
Clinical outcome	1.000	1.000	1.000	1.000	1.000										
CPG	0.845	2.112	0.907	0.831	-0.092	0.911									
Financial outcome	-5.231	0.868	0.704	0.860	0.672	-0.128	0.928								
Nurse adequacy	1.000	1.000	1.000	1.000	0.004	0.006	-0.085	1.000							
Pandemic status	1.000	1.000	1.000	1.000	-0.002	-0.006	0.089	-0.621	1.000						
Pandemic∗CPG (CO)	1.000	1.000	1.000	1.000	-0.018	-0.018	-0.033	0.005	-0.003	1.000					
Pandemic∗CPG (FO)	1.000	1.000	1.000	1.000	-0.018	-0.018	-0.033	0.005	-0.003	1.000	1.000				
Pandemic∗ supervision (CO)	1.000	1.000	1.000	1.000	0.020	0.005	-0.034	0.039	-0.047	-0.011	-0.011	1.000			
Pandemic∗supervision (FO)	1.000	1.000	1.000	1.000	0.020	0.005	-0.034	0.039	-0.047	-0.011	-0.011	1.000	1.000		
Patient's condition	0.678	0.792	0.854	0.747	0.468	-0.032	0.286	-0.030	0.069	-0.025	-0.025	-0.028	-0.028	0.864	
Supervision	0.974	0.985	0.987	0.975	-0.004	-0.013	-0.163	0.122	-0.088	0.006	0.006	0.078	0.078	0.213	0.987

Note: CPG = clinical practice guidelines; CO = clinical outcome; FO = financial outcome.

**Table 4:** Heterotrait–Monotrait Ratio (HTMT).

Constructs	Clinical outcome	ClPG	Financial outcome	Nurse adequacy	Pandemic status	Pandemic∗CPG (CO)	Pandemic∗CPG (FO)	Pandemic∗supervision (CO)	Pandemic∗supervision (FO)	Patient's condition
Clinical outcome										
Clinical practice guidelines	0.085									
Financial outcome	0.726	0.113								
Nurse adequacy	0.004	0.009	0.091							
Pandemic status	0.002	0.012	0.098	0.621						
Pandemic∗CPG (CO)	0.018	0.020	0.036	0.005	0.003					
Pandemic∗CPG (FO)	0.018	0.020	0.036	0.005	0.003	1.000				
Pandemic∗supervision (CO)	0.020	0.008	0.037	0.039	0.047	0.011	0.011			
Pandemic∗supervision (FO)	0.020	0.008	0.037	0.039	0.047	0.011	0.011	1.000		
Patient's condition	0.539	0.153	0.327	0.035	0.081	0.030	0.030	0.032	0.032	
Supervision	0.004	0.040	0.177	0.124	0.086	0.006	0.006	0.079	0.079	0.279

Note: CPG = clinical practice guidelines; CO = clinical outcome; FO = financial outcome; aLOS = average length of stay.

**Table 5:** Cross loadings.

Constructs	Pandemic status	Patient's condition	Clinical practice guidelines	Supervision	Nurse adequacy	Clinical outcome	Financial outcome	Pandemic∗CPG (CO)	Pandemic∗supervision (CO)	Pandemic∗CPG (FO)	Pandemic∗supervision (FO)
Pandemic status	1.000	0.069	-0.006	-0.088	-0.621	-0.002	0.089	-0.003	-0.047	-0.003	-0.047
Severity	0.046	0.929	-0.088	0.239	-0.021	0.283	0.119	-0.018	-0.017	-0.018	-0.017
Complexity	0.070	0.794	0.008	0.155	-0.029	0.488	0.332	-0.025	-0.029	-0.025	-0.029
CPG_percent_coverage	0.010	-0.148	0.988	-0.066	-0.007	-0.046	-0.027	-0.016	0.009	-0.016	0.009
CPG_compliance	-0.010	0.001	0.827	0.002	0.009	-0.099	-0.148	-0.017	0.004	-0.017	0.004
Supervisor_availability	-0.124	0.210	-0.013	0.986	0.125	-0.007	-0.165	0.004	0.091	0.004	0.091
Supervision_method	-0.044	0.210	-0.014	0.989	0.117	-0.001	-0.157	0.007	0.062	0.007	0.062
Nurse_adequacy	-0.621	-0.030	0.006	0.122	1.000	0.004	-0.085	0.005	0.039	0.005	0.039
aLOS	-0.002	0.468	-0.092	-0.004	0.004	1.000	0.672	-0.018	0.020	-0.018	0.020
Total_cost_of_care	0.078	0.367	-0.102	-0.179	-0.089	0.685	0.944	-0.033	-0.036	-0.033	-0.036
Claim profit	-0.089	-0.141	0.140	0.119	0.066	-0.549	-0.911	0.027	0.027	0.027	0.027
Pandemic status ∗ clinical practice guidelines (CO)	-0.003	-0.025	-0.018	0.006	0.005	-0.018	-0.033	1.000	-0.011	1.000	-0.011
Pandemic status ∗ supervision (CO)	-0.047	-0.028	0.005	0.078	0.039	0.020	-0.034	-0.011	1.000	-0.011	1.000
Pandemic status ∗ clinical practice guidelines (FO)	-0.003	-0.025	-0.018	0.006	0.005	-0.018	-0.033	1.000	-0.011	1.000	-0.011
Pandemic status ∗ supervision (FO)	-0.047	-0.028	0.005	0.078	0.039	0.020	-0.034	-0.011	1.000	-0.011	1.000

Note: CPG = clinical practice guidelines; CO = clinical outcome; FO = financial outcome.

**Table 6:** Collinearity statistics (VIF) inner VIF values.

Constructs	Patient's condition	Clinical practice guidelines	Supervision	Nurse adequacy	Clinical outcome	Financial outcome
Pandemic status	1.000	1.000	1.005	1.000	1.638	1.640
Patient's condition			1.005		1.060	1.381
Clinical practice guidelines					1.001	1.010
Supervision					1.074	1.093
Nurse adequacy					1.641	1.641
Clinical outcome						1.315
Financial outcome						
Pandemic∗CPG (CO)					1.001	
Pandemic∗supervision (CO)					1.010	
Pandemic∗CPG (FO)						1.001
Pandemic∗supervision (FO)						1.012

Note: CPG = clinical practice guidelines; CO = clinical outcome; FO = financial outcome.

**Table 7:** Path coefficients, mean, SD, *T* values, *P* values, and decision of hypotheses.

Hypotheses	Path	Beta	Mean	SD	*T* values	*P* values	95% CI	Decision
1	Pandemic status ⟶ clinical outcome	-0.041	-0.041	0.006	6.786	0.000	-0.054 to -0.030	Supported
2	Pandemic status ⟶ financial outcome	0.055	0.055	0.006	9.839	0.000	0.044 to 0.065	Supported
3	Pandemic status ⟶ patient's condition	0.069	0.070	0.006	12.421	0.000	0.058 to 0.080	Supported
4	Pandemic status ⟶ nurse adequacy	-0.621	-0.621	0.004	139.974	0.000	-0.631 to -0.613	Supported
5	Pandemic status ⟶ supervision	-0.103	-0.102	0.005	19.314	0.000	-0.113 to -0.092	Supported
6	Pandemic status ⟶ clinical practice guidelines	-0.006	-0.006	0.005	1.123	0.262	-0.017 to 0.004	Rejected
7	Patient's condition ⟶ supervision	0.220	0.220	0.005	46.335	0.000	0.211 to 0.229	Supported
8	Supervision ⟶ clinical outcome	-0.118	-0.118	0.005	24.855	0.000	-0.128 to -0.109	Supported
9	Supervision ⟶ financial outcome	-0.150	-0.151	0.007	21.976	0.000	-0.163 to -0.136	Supported
10	Clinical practice guidelines ⟶ clinical outcome	-0.078	-0.078	0.003	24.550	0.000	-0.084 to -0.072	Supported
11	Clinical practice guidelines ⟶ financial outcome	-0.069	-0.069	0.004	19.508	0.000	-0.076 to -0.062	Supported
12	Patient's condition ⟶ clinical outcome	0.494	0.494	0.006	86.868	0.000	0.482 to 0.506	Supported
13	Patient's condition ⟶ financial outcome	-0.002	-0.001	0.007	0.263	0.793	-0.015 to 0.010	Rejected
14	Nurse adequacy ⟶ clinical outcome	0.007	0.007	0.006	1.145	0.253	-0.004 to 0.018	Rejected
15	Nurse adequacy ⟶ financial outcome	-0.034	-0.033	0.007	4.737	0.000	-0.047 to -0.020	Supported
16	Clinical outcome ⟶ financial outcome	0.667	0.666	0.019	34.340	0.000	0.622 to 0.699	Supported
17	Pandemic∗ CPG (CO) ⟶ clinical outcome	-0.006	-0.006	0.003	1.735	0.083	-0.012 to 0.001	Rejected
18	Pandemic∗supervision (CO) ⟶ clinical outcome	0.040	0.041	0.005	8.825	0.000	0.032 to 0.049	Supported
19	Pandemic∗CPG (FO) ⟶ financial outcome	-0.022	-0.022	0.002	9.376	0.000	-0.027 to -0.017	Supported
20	Pandemic∗supervision(FO) ⟶ financial outcome	-0.031	-0.031	0.005	6.386	0.000	-0.041 to-0.023	Supported

Note: CPG = clinical practice guidelines; CO = clinical outcome; FO = financial outcome.

**Table 8:** Discriminant validity *R* square, *f* square, and *Q* square.

Constructs	*R* ^2^ adjusted	*Q* ^2^	*f* ^2^					
			Clinical outcome	Clinical practice guidelines	Financial outcome	Nurse adequacy	Patient condition	Supervision
Clinical outcome	0.240	0.238	0.240		0.663			
Clinical practice guidelines	0.000	0.000	0.000		0.009			
Financial outcome	0.490	0.413	0.490					
Nurse adequacy	0.386	0.384	0.386		0.001			
Pandemic status			0.001	0.000	0.004	0.628	0.005	0.011
Pandemic∗CPG (CO)			0.000					
Pandemic∗CPG (FO)					0.001			
Pandemic∗supervision (CO)			0.002					
Pandemic∗*s*upervision (FO)					0.002			
Patient's condition	0.005	0.003	0.303		0.000			0.051
Supervision	0.056	0.054	0.017		0.040			

Note: CPG = clinical practice guidelines; CO = clinical outcome; FO = financial outcome.

## Data Availability

The authors confirm that the data supporting the findings of this study are available within the article.
